This article has been retracted.

# Study on the Cytotoxic Microstructure of Titanium Dioxide Nanoparticles by X-Ray Phase-Contrast CT Imaging

**DOI:** 10.1155/2022/2413922

**Published:** 2022-07-30

**Authors:** Jingtong Fei, Shanshan Nie, Bo Zhang, Xinli Teng, Ying Chen, Yikun Qu, Zhuoxin Cheng, Linqi Guo

**Affiliations:** ^1^The First Affiliated Hospital of Jiamusi University, Intensive Care Unit, Jia Mu Si 154000, China; ^2^Jiamusi University, Department of Pathophysiology, Jia Mu Si 154000, China; ^3^The Tumor Hospital of Jiamusi, Department of Tumor, Jia Mu Si 154000, China; ^4^The First Affiliated Hospital of Jiamusi University, Department of General Surgery, Jia Mu Si 154000, China

## Abstract

To address the problem of microstructural analysis of titania nanoparticles with high cytotoxicity, the authors propose X-ray phase-comparative CT imaging studies. In this method, the HE-stained section samples were compared with the X-ray phase-contrast CT imaging microscopic images, and 3D texture analysis was used to observe the changes in the preparation of hepatocyte microstructures in the two groups. The results show that X-ray phase-contrast CT imaging microscopic images and their larger image size are closely related to HE staining images, and X-ray phase-contrast CT microscopic images can observe important data of hepatocytes from multiple angles. The ship skeleton extraction method based on the endpoint limit also has advantages over traditional algorithms in extraction accuracy and can provide more 3D feature files, confirming the growth and transformation of normal hepatocytes into hepatocyte cytotoxic microstructures. The distribution effect of using the ensemble process is better than the simple 2D feature set and 3D feature set, and the overall accuracy is improved; the result distribution of the tree determination and random forest methods is also better than that of the support vector machine method. The experimental results show that the X-ray phase-contrast CT images can highlight the 2D and 3D imaging features of the hepatotoxic microstructure of TiO_2_ nanoparticles and provide data for quantitative analysis.

## 1. Introduction

Titanium dioxide (TiO_2_) is a nontoxic material with anticorrosion and photochemical catalytic properties and is widely used in the fields of medicine, daily medicine, cosmetics, and food. Studies have shown that it can enter the human body through respiration and digestion and is particularly effective, thereby causing toxicity to the body [1]. It is often precipitated in the liver. With the increase of the concentration, liver function is significantly damaged, and a series of syndromes such as the antioxidant system, immune dysfunction, and systemic inflammatory response are caused [2]. X-ray phase-contrast imaging (PCI) typically utilizes a phase shift from the previous X-ray image model to obtain contrast images. Compared with conventional X-ray, the contrast of the contrast image is very good, and the soft cell model image at the micron or even submicron scale can be seen. Combined with PCI and tomography (e.g., tomography and CT), comparative CT can present high-resolution three-dimensional (3-dimensional, 3D) images of the internal model of the model [3]. Early detection of hepatotoxicity typically involves the use of diagnostic imaging, molecular marker testing, and protein marker testing. In adult screening, screening is an easier and faster way. A combination of differential-based X-ray imaging techniques has been widely used in medicine, biology, data science, data science, and various applications [4]. The application characteristics of X-ray phase-comparison CT imaging, microscopic imaging of liver diseases, and the structure of liver toxicity are explored, in order to effectively promote the application and development of X-ray phase-comparison CT imaging technology in the field of biomedicine, as shown in Figure 1.

## 2. Literature Review

Since scientists discovered X-rays, X-ray imaging has become a widely used diagnostic tool. The most commonly used imaging techniques (such as conventional X-ray, ultrasound, and MRI) are limited by their graphic design and cannot meet the requirements of hepatotoxicity microscopic imaging in terms of comparison and resolution [2]. X-ray phase-contrast CT is based on X-rays passing through the model, and the data stage carries the images in the model, solving the problem of soft tissue microscopic images with new images [5].

Singer et al. developed an X-ray interferometer containing three equivalent Laue crystals, which made it possible to record different levels of X-rays refracted by the material [6]. Kumar et al. found that X-ray grating phase comparison images do not use the Talbot effect, but are based on geometric projection patterns with an optical design similar to the Talbot-Lau interferometer [7]. Vila-Comamala proposed a fast, low-dose ECG raster CT reconstruction algorithm called the back-projection algorithm [8]. Zhou' research is on dynamic grating imaging using high-throughput polychromatic illumination and a fixed grating imaging system [9]. Kalasova asked to reduce the number of steps, so that only the images obtained from a part of the work intersected with the data of the important work obtained by the intervention, which also achieved the purpose of reducing the exposure time [10]. Zverev devised a method for acquiring interlaced grating phase-similar CT data that enables the data to be obtained similar to the process of grating phase-comparison CT for conventional CT imaging, speeding up the imaging process and reducing radiation dose [11].

Based on the current study, the authors announce a study of X-ray phase-contrast CT images. X-ray equipment offers the ability to refine new image formats based on differences in the interaction of X-rays with images and features of the product compared to traditional image formats, and it can make images through the identification stage. The coefficient of the X-ray after passing through the material, for weakly absorbing materials, the phase coefficient of the material which is several times the absorption coefficient, and images with higher spatial resolution and contrast can be obtained [12]. It can be used to observe highly cytotoxic models, and X-ray phase-contrast CT imaging has also become one of the most advanced technologies and research hotspots.

## 3. X-Ray Phase-Contrast CT Imaging Principle

### 3.1. Synchrotron Radiation

Synchrotron radiation (SR) was first discovered at a synchrotron; this is also the origin of its name; it means that electrons move in a curved line at a speed close to the speed of light in a magnetic field, a type of electromagnetic radiation emitted in a tangential direction [13]. Early synchrotron radiation was not favored by high-energy physicists because its existence has caused great damage to the energy, which in turn affects the improvement of the energy of the high-energy accelerator; it is a factor that must be excluded. Later, scientists found that synchrotron radiation has high coherence, high collimation, wide spectral range, and other excellent performances that conventional light sources cannot match. The excellent characteristics of synchrotron radiation have brought broad prospects for the development of related scientific and applied research [14].

The synchrotron radiation source is a generator of synchrotron radiation, and it has experienced three generations of rapid development since its birth. The first generation light source is a dual-purpose machine for high-energy colliders, the second generation light source is a dedicated machine based on a dedicated storage ring for synchrotron radiation, and the third generation light source is based on a dedicated machine with a higher performance synchrotron radiation dedicated storage ring [15].

Synchrotron radiation light source has very excellent characteristics, and its main characteristics are as follows:

1. High brightness: The radiation power is very high, which is hundreds of millions of times that of conventional light sources (such as X-ray machines). Synchrotron radiation can complete a picture of crystal defects in more than ten seconds.
2. Broadband: A continuous spectrum from infrared to X-ray, a specific wavelength of light can be obtained using a monochromator.
3. High collimation: Almost collimated light. Trace elements in materials or very small samples can be studied.
4. High polarization: Linear polarization, circular/elliptical polarization can be achieved.
5. High purity: No pollution, spectrum can be calculated accurately.

Synchrotron radiation light sources also have the characteristics of narrow pulse and high coherence, which make it possible for synchrotron radiation to be applied to high-resolution and high-contrast biomedical imaging.

### 3.2. X-Ray Phase-Contrast CT Imaging and Its Physical Principles

The initial X-ray imaging is mainly based on the projection of the sample in a certain direction, the structural information inside the sample is superimposed on the X-ray propagation direction, and the spatial relationship and specific structure cannot be distinguished before and after [16]. Computed tomography, or CT, measures the sample by projecting it from different angles; furthermore, the imaging technology that obtains the cross-sectional information of the sample through the reconstruction algorithm, combined with the three-dimensional visualization technology, can reveal the internal information of the sample and its three-dimensional structure.

Since the first prototype of X-ray CT imaging was developed, the model has immediately caused a huge response in the medical community, which has led to the rapid development of CT imaging technology, which consumes less energy. Traditional CT imaging usually relies on the information attenuation of X-rays passing through the equipment. Different equipment cause different attenuations of X-rays. The X-ray output will carry internal vacuum data. Product vacuum data can be picked up by detectors and then converted into images of the material's internal structure, known as X-ray absorption CT. However, the X-ray reduction of light structures such as soft tissues of the body is small, making it difficult to obtain sufficient contrast for CT scanning [17]. X-ray phase comparison is based on the phase data carried by X-rays after passing through the sample and has achieved excellent results in the field of cell image processing. Early contrast studies were often based on projected images, which limited the development of the contrast stage.

In recent years, with the combination of phase-contrast and CT technology, namely, phase-contrast CT, phase-contrast imaging has been developed and applied more and more. Phase-contrast CT has the advantages of phase difference and CT quality. It can not only analyze the detailed data in the model but also combine with 3D reconstruction algorithms. Phase-contrast CT can also obtain three-dimensional modeling, which can analyze the details in the model. The internal structure of the model is observed from any angle, and the triangular model of a certain model is observed multiple times [18]. In addition, with the rapid development of third generation synchrotron imaging equipment such as lighting equipment, CT contrast phase has received more attention and has become a research hotspot in the field of biomedical imaging.

### 3.3. X-Ray Phase-Contrast Imaging Characteristics

Different devices have different attenuation rates for X-rays, which is important for X-ray imaging, which is the principle of X-ray imaging by evaluating the difference in the transit time of X-rays through solids. Look at the internal structure of the object [19]. The study found that the decay of X-rays in an object is related to the amount of matter, which is easier to place, and the decay rate increases with speed. The human cell structure formed by different elements can only be based on art, and its density can be divided into three groups: high-density bone cells and calcification foci; middle cartilage, connective tissue and muscle; and ovary and tooth decay. It plays a key role in the third stage of the X-ray imaging system, receiving the X-ray residue after passing through the body through the X-ray detector and performing the X-ray procedure to create the image, as shown in Figure 2.

## 4. Experiments and Research

### 4.1. Evaluation of the Extraction Effect

To calculate the accuracy of the extraction results, the analysis was performed using mean (AD) and true (CR) measurements, which refer to the mean of the bones. Subtract the intermediate design value and the true value. It refers to the proportion of the bones extracted from the average model [20]. The coronary arteries of mice were extracted using two methods, the median artery was extracted, and the mean distance and accuracy were calculated, and the medial centerline vessels subtracted from the improvement were less than this value when examining the samples. The actual cost of the traditional “electric way” is also increasing.

### 4.2. 3D Vascular Network Analysis

Three-dimensional vascular body density (MVD-3D) refers to the proportion of the volume occupied by blood vessels per unit volume; it reflects the density of blood vessels in a certain spatial area and is also a parameter index describing the distribution of blood vessels [21]. After calculation, the average volume density of three-dimensional blood vessels of normal, diffuse, proliferative, and irregular cystic hepatotoxicity microstructures was obtained, there was no significant difference in the density of three-dimensional vascular bodies between normal and diffuse types, there were statistically significant differences between the normal group and the other types of three-dimensional vascular body density, and the differences between the diffuse type and the other two types of three-dimensional vascular body density were also statistically significant.

Perform frequency distribution statistics on blood vessels of different diameters and record the data of the main distribution results of blood vessel diameters in normal liver cells. Diffuse hepatotoxicity microstructural vessel diameter main distribution results record data. The main distribution results of the vascular diameter of the microstructure of proliferative diffuse hepatotoxicity were recorded data. The results showed that the vascular diameter of cells with irregular hepatotoxicity microstructure was generally larger, and the difference was statistically significant; it was distributed in all diameters, and some vascular diameters even reached high grades [22].

### 4.3. 2D Image Feature Extraction of Hepatocyte Microstructure

This part of the study extracted two-dimensional X-ray phase-contrast CT images of normal, diffuse, proliferative, and irregular cystic hepatotoxicity microstructures and calculated five types of eigenvalues of the selected images, including grayscale histogram, grayscale co-occurrence matrix, gray-gradient co-occurrence matrix, Tamura texture, and wavelet transform [23]. Calculate the time consumed by each feature algorithm, the time required to extract gray histogram features is the shortest, and the extraction time of normal images is also shorter than that of other types of images. It takes the longest time to extract physical features of Tamura, and the extraction time of normal images is also shorter than that of other types of images, and the difference is statistically significant. For different types of images, the extraction time of the normal type is also shorter than that of other types.

### 4.4. Classification Results of Hepatocyte Microstructure

To differentiate hepatotoxic microstructure from normal hepatocyte images, the authors provided 2D and 3D features, feature selection, and analysis classification studies from data from various hepatotoxic microstructure specimens and normal hepatocyte microstructure specimens [24]. For image extraction, PCA and AUC area constraints were used for screening and size reduction, and the process we completed was separated by C4.5 tree determination, random valley, forest, and support vector techniques. A 10-fold cross-validation method was used to classify among the three classifiers. For X-ray phase-contrast CT imaging microscopic images, in each round of standard validation, a subset model was randomly selected according to the training model. The set is used to train the model, and the process is used as the test set to validate the model.

## 5. Results and Analysis

Using C4.5 decision tree, random forest, and support vector machine methods to classify and identify the three-dimensional feature set, the C4.5 decision tree method was used to calculate the accuracy of the classification of normal, diffuse, proliferative, and irregular hepatotoxic microstructure specimens. Accuracy calculation of the classification of normal, diffuse, proliferative, and irregular hepatotoxic microstructure specimens was done using random forest methods. The classification accuracy of normal type, diffuse type, proliferative type, and irregular hepatotoxicity microstructure specimens was calculated by using the support vector machine method. The classification results obtained are compared.

C4.5 decision tree, random forest, and support vector machine methods were used to classify and identify two-dimensional feature sets, respectively, and the C4.5 decision tree method was used to classify normal, diffuse, proliferative, and irregular hepatotoxic microstructure specimens. The random forest method was used to calculate the classification accuracy of normal, diffuse, proliferative and irregular hepatotoxic microstructure specimens. The accuracy of the classification of normal, diffuse, proliferative, and irregular hepatotoxic microstructure specimens using the support vector machine method was calculated separately.

The C4.5 decision tree, random forest and support vector machine methods were used to classify and identify the two-dimensional and three-dimensional mixed feature sets, and the C4.5 decision tree method was used to classify the normal, diffuse, proliferative, and irregular hepatocyte toxicity microstructures, and the accuracy of specimen classification is calculated. The random forest method was used to calculate the classification accuracy of normal, diffuse, proliferative, and irregular hepatotoxic microstructure specimens. The accuracy of the classification of normal, diffuse, proliferative, and irregular hepatotoxic microstructure specimens was calculated using the support vector machine method.

The results show that the classification effect of the mixed feature set is better than that of the simple two-dimensional feature set and the three-dimensional feature set, and the overall result is improved. The classification effect of the decision tree and random forest method is also better than that of the support vector machine method. Experimental results show X-ray phase-contrast CT imaging can clearly display the 2D and 3D image features of the hepatotoxic microstructure of TiO_2_ nanoparticles and provide a reference for the quantitative analysis of their structures.

## 6. Discussion

Focusing on the requirements of tertiary prevention and precision medicine, the authors used X-ray phase-contrast CT imaging to image normal hepatocytes and diffuse, proliferative, and irregular hepatocyte cytotoxic microstructures, the three-dimensional vascular network was reconstructed and then skeletonized and quantitatively analyzed; extract three-dimensional quantitative features and quantitative features of two-dimensional images and use the area under the ROC curve method and PCA principal component analysis method to screen and reduce the dimension of high-dimensional feature quantities; finally, a machine learning algorithm is applied to classify the optimized feature set and evaluate the classification effect. Explore the application of vascular skeletonization analysis and machine learning methods in the study of hepatocyte classification and prediction and provide clinicians with a more meaningful solution for auxiliary diagnosis to detect liver diseases as soon as possible.

## 7. Conclusion

Biosafety is a prerequisite for the use of nanomaterials such as TiO_2_ nanoparticles in the field of biomedical engineering. Much is now known about the negative effects of titanium dioxide nanoparticles on hepatocytes. Entering into human tissue or coming into contact with the human body, the role of both and the human body is a complex process that requires a deep understanding of their relationship and meaning. The advent of synchrotron X-ray sources, especially polar colliding monochromatic X-ray sources with constant tunable wavelengths, has opened up the possibility of improving new photographs. Compared with conventional X-ray absorption contrast imaging, MRI, and other imaging techniques such as ultrasound imaging, X-ray phase-contrast CT imaging shows good results for high-resolution microscopic imaging of tissues and can perform high-precision microscopic imaging, 3D visualization. The X-ray phase-contrast CT imaging method has a wide range of application value in the field of biomedicine. This is particularly important for early detection, early diagnosis, and early treatment proposed for tertiary disease prevention.

## Figures and Tables

**Figure 1:** Titanium dioxide nanoparticles.

**Figure 2:** X-ray phase-contrast imaging characteristics.

## Data Availability

The data used to support the findings of this study are available from the corresponding author upon request.
